RETRACTED

# MiR-200b regulates autophagy associated with chemoresistance in human lung adenocarcinoma

**DOI:** 10.18632/oncotarget.5352

**Published:** 2015-09-21

**Authors:** Banzhou Pan, Bing Feng, Yitian Chen, Guichun Huang, Rui Wang, Longbang Chen, Haizhu Song

**Affiliations:** ^1^ Department of Medical Oncology, Jinling Hospital, School of Medicine, Nanjing University, Nanjing 210002, China

**Keywords:** miR-200b, autophagy, chemoresistance, human lung adenocarcinoma, ATG12

## Abstract

Chemoresistance remains a major clinical problem in combating human lung adenocarcinoma (LAD), and abnormal autophagy is closely associated with this phenomenon. In the present study, an inverse correlation between miR-200b and autophagy-associated gene 12 (ATG12) expressions was observed in docetaxel-resistant (SPC-A1/DTX and H1299/DTX) and sensitive (SPC-A1 and H1299) LAD cells as well as in tissue samples. Further study showed that miR-200b directly targeted ATG12 in LAD. Moreover, miR-200b-dependent ATG12 downregulation inhibited autophagy and enhanced the chemosensitivity of SPC-A1/DTX and H1299/DTX cells both *in vivo* and *in vitro*. LAD chemoresistance is therefore closely related to downregulation of miR-200b and the corresponding upregulation of ATG12. These results provide new evidence for the mechanisms governing the microRNA (miRNA)-ATG12 network and their possible contribution to autophagy modulation and LAD chemoresistance.

## INTRODUCTION

Non-small-cell lung cancer (NSCLC) accounts for approximately 80% of all lung cancers and is the leading cause of cancer-related deaths worldwide [1, 2]. NSCLC is the most common histological type of LAD. Current standard treatments for LAD include surgical resection, platinum-based chemotherapy, radiation therapy or a combination of these methods. Unfortunately, LAD has a poor prognosis and rapidly develops resistance to antineoplastic drugs both *in vivo* and *in vitro* [3]. Patients with resistant disease, especially at an advanced stage, suffer early relapse with an overall 5 year survival rate of only 15% [2]. Identifying the underlying mechanisms of LAD chemoresistance is therefore of major importance in the clinical application of chemotherapy.

Autophagy is an evolutionarily conserved process responsible for intracellular degradation of long-lived proteins and organelles [4]. Autophagy is rapidly activated in response to intracellular (e.g. accumulation of unfolded proteins, damaged or surplus organelles, pathogens) and extracellular (e.g. starvation, hypoxia) stress factors and provides recycled metabolic substrates necessary for survival [5]. Through the concerted action of several protein complexes (consisting of a number of conserved autophagy-related proteins), double-membrane vesicles called autophagosome are produced that transport cytoplasmic components into lysosomes for degradation [6, 7]. Among autophagy-related proteins, there are two classes of ubiquitin-like proteins: the autophagy-related MAP1LC3 (LC3) family (which consists of seven members in mammals) and ATG12, which share some sequence similarities [8]. LC3 and ATG12 are activated by the same E1-like enzyme ATG7, and subsequently transferred to the E2-like enzymes, ATG3 and ATG10, respectively. ATG3 conjugates ATG8 to the membrane lipid phosphatidylethanolamine (PE) at autophagosome-forming sites, where this conjugate recruits cytoplasmic cargo and assists expansion of the isolation membrane [9]. However, ATG10 attaches ATG12 to another structural protein, ATG5, which results in the eventual formation of the ATG12-ATG5-ATG16 complex. This complex acts as an E3-like enzyme to facilitate ATG8-PE formation [10]. Indeed, cells lacking any of the conjugation reaction components exhibit autophagy defects.

RETRACTED

Although certain studies regard autophagy as an alternative form of stress-induced cell death, overwhelming evidence supports the idea that autophagy functions primarily as a pro-survival mechanism, which leads to chemoresistance [11]. We previously reported that LAD cells use autophagy to evade antitumor drugs; mechanistic investigation revealed that HMGB1 triggers autophagy by promoting Beclin-1-PI3K-III core complex formation through activation of the MEK/ERK1/2 signaling pathway [12]. Nevertheless, despite advances in our understanding of the process of autophagy, the mechanisms regulating this multi-stage process remain largely unknown. Considering the importance of both miRNAs and autophagy in cancer-related processes [13], and given the lack of strong evidence linking these two rapidly growing fields of research in LAD, here we investigate the role of miRNAs in autophagy.

MiRNAs are small non-coding RNAs that post-transcriptionally regulate gene expression by base paring with specific mRNA target sequences (mainly 3′-untranslated regions (3′-UTR)), which leads to translational inhibition or mRNA degradation [14]. A growing number of miRNAs reportedly regulate the expression of ATG genes, or their regulators, at different autophagy steps [15]. However, the mechanism whereby dysregulated miRNAs affect autophagic activity in chemoresistant NSCLC cells remains poorly understood.

Herein, we report that miR-200b, a down-regulated miRNA in docetaxel-resistant LAD cells, remarkably inhibits autophagy activation and enhances sensitivity to multiple antitumor drugs. Specifically, we report for the first time that *ATG12* is a direct target of miR-200b in LAD. We demonstrate miR-200b-dependent downregulation of *ATG12*, which blocks autophagy and resensitized LAD cells to chemotherapy both *in vivo* and *in vitro*. Our study confirms the importance of miRNAs in autophagy control and provides the first evidence for miR-200b-dependent regulation of autophagy.

RETRACTED

## RESULTS

### Forced expression of miR-200b blocks autophagy in LAD cells

We previously demonstrated that autophagy acts as a resistance mechanism in docetaxel-resistant SPC-A1/DTX cells and that suppression of high-mobility group box 1 (HMGB1) or limiting HMGB1 cytosolic translocation alleviated autophagic protection in response to docetaxel [12]. Here we were interested to explore the role of miRNAs in the development of autophagy-related docetaxel resistance in LAD cells.

Using microarrays, we previously showed that 6 of 52 miRNAs were differentially expressed more than two fold in docetaxel-resistant SPC-A1/DTX cells compared with parental SPC-A1 cells, including three upregulated miRNAs (miR-192, miR-424 and miR-98) and three downregulated miRNAs (miR-200b, miR-194 and miR-212) [16]. The qRT-PCR data reported here was consistent with our previously reported microarray results, confirming their validity (Supplementary Fig. 1A). We hypothesized that these dysregulated miRNAs contribute to increased autophagy in SPC-A1/DTX cells. To test our hypothesis, we transfected sequence-specific inhibitors of upregulated miRNAs or precursors of downregulated miRNAs into SPC-A1/DTX cells and then detected the incidence of autophagy; an increased LC3-II/LC3-I ratio was considered evidence for autophagy induction [17]. Western blot analysis demonstrated that, compared with a nonspecific mimic or inhibitor-negative control, the miR-200b mimic (PmiR-200b) exhibited maximum inhibitory potency against autophagy activity, as demonstrated by the significant decrease in the conversion of LC3-I to LC3-II (Fig. 1A). We therefore selected miR-200b to further explore the influence of miRNAs on autophagy.

**Figure 1:** Forced expression of miR-200b blocks autophagy in SPC-A1/DTX cells **A.** SPC-A1/DTX cells were transfected with the indicated miRNA precursors. Whole cell lysates were analyzed by western blot for LC3-II/LC3-I protein. LC3-II/LC3-I and LC3-II/GAPDH ratios were calculated by Image J densitometric analysis (three independent experiments gave similar results). **B.** Docetaxel-resistant SPC-A1/DTX cells transfected with PmiR-200b and parental SPC-A1 cells transfected with AmiR-200b were exposed to docetaxel (100 μg/L and 10 μg/L, respectively) and cisplatin (1.5 μg/ml and 0.5 μg/ml, respectively) for 48 h. Whole cell lysates were analyzed by western blot using LC3 and P62 antibodies (control: GAPDH). LC3-II/LC3-I and P62/GAPDH ratios were calculated using Image J densitometric analysis (three independent experiments gave similar results). **C.** SPC-A1/DTX cells and SPC-A1 cells were transfected with a GFP-LC3 construct and either PmiR-200b or AmiR-200b, following treatment with docetaxel (100 μg/L and 10 μg/L, respectively) or cisplatin (1.5 μg/ml and 0.5 μg/ml, respectively). GFP-LC3 dot formation was analyzed as described in the Materials and Methods section (bar: 50 μm). The results are presented as mean ± SD of values obtained in three independent experiments. *P < 0.05; **P < 0.01. **D.** SPC-A1 cells were transfected with AmiR-NC or AmiR-200b for 48 h. Cell samples were prepared for transmission electron microscopy analysis. Arrows indicate autophagosomes. N: nucleus. **E.** SPC-A1/DTX cells transfected with PmiR-200b were treated with docetaxel (100 μg/L) after incubation with Baf A1 (20 nM) for 2 h or not. SPC-A1 cells transfected with AmiR-200b were treated with Baf A1 (20 nM, 2 h) or not. Cell lysates were analyzed by western blot for LC3 and P62 (control: GAPDH). LC3-II/GAPDH and P62/GAPDH ratios were calculated using Image J densitometric analysis (three independent experiments gave similar results). **F.** Western blot analysis for LC3, P62 and ATG5 in SPC-A1 cells co-transfected with AmiR-200b and ATG5 siRNA. LC3-II/LC3-I and P62/GAPDH ratios were calculated using Image J densitometric analysis (three independent experiments gave similar results).

RETRACTED

SPC-A1/DTX cells with a relatively higher LC3-II/LC3-I ratio were transfected with PmiR-200b to upregulate miR-200b expression. Ectopic miR-200b attenuated the conversion of LC3-II to LC3-I and prevented P62 degradation with or without treatment with docetaxel or cisplatin (Fig. 1B). Additionally miR-200b-dependent inhibition of autophagy was confirmed by GFP-LC3 fluorescence microscopy, where the percentage of punctate GFP^+^ SPC-A1/DTX cells was reduced (Fig. 1C). In contrast, suppressing miR-200b (by transfecting a miR-200b inhibitor (AmiR-200b) into SPC-A1 cells) resulted in elevated turnover of LC3-II and increased the percentage of punctate GFP-positive cells (Fig. 1B, 1C). The formation of characteristic autophagosomes further confirmed the increased autophagic activity, as observed by transmission electron microscopy (Fig. 1D).

Diminished LC3-II levels can be caused by blocking autophagosome formation or by excessive clearance of autophagosomes. To distinguish between these two possibilities, Bafilomycin A1 (Baf A1), which blocks autophagosome-lysosome fusion, was employed to prevent LC3-II degradation [18]. Following docetaxel treatment, LC3-II accumulation was further enhanced in Baf A1-pretreated control SPC-A1/DTX cells, but only minimally altered in miR-200b-transfected cells (Fig. 1E). Conversely, LC3-II accumulation was not affected by Baf A1 when administering AmiR-200b, suggesting that the increased in LC3-II was caused by autophagy induction as opposed to inhibition of autophagosome clearance mediated by miR-200b (Fig. 1E). Furthermore, blocking autophagy with ATG5 siRNA abolished AmiR-200b-dependent formation of LC3-II (Fig. 1F).

RETRACTED

To extend our findings, we prepared another docetaxel-resistant LAD cell line, H1299/DTX, from docetaxel-sensitive H1299 cells *in vitro*. H1299/DTX cells exhibited a 2.81-fold downregulation in miR-200b expression compared with parental H1299 cells (Supplementary Fig. 1B). Similar to the results in SPC-A1/DTX cells, forced expression of miR-200b limited autophagy activity in H1299/DTX cells even when treated with cytotoxic agents, as shown by diminished LC3-II/LC3-I ratios and the reduction in punctate GFP-positive cells (Supplementary Fig. 2A, 2B). By contrast, miR-200b silencing led to the activation of autophagy, which was further enhanced when exposed to antitumor drugs (Supplementary Fig. 2A, 2B). Meanwhile, AmiR-200b transfection into H1299 cells resulted in LC3-II accumulation, whereas Baf A1 pretreatment failed to further increase LC3-II accumulation (Supplementary Fig. 2C). Collectively, these data indicate that miR-200b negatively regulates autophagy in LAD cells.

### MiR-200b suppresses autophagy by directly targeting ATG12

To further investigate the mechanisms of miR-200b-dependent inhibition of autophagy, we sought to identify putative autophagy-related targets of miR-200b, based on the miRNA database(http://microRNA.org). The miR-200b seed sequence matched nucleotides in the *ATG12* sequence (Fig. 2A). Furthermore, using a dual-luciferase reporter system we demonstrated that miR-200b binds directly to the 3′UTR of *ATG12* mRNA. This was done by cloning full-length *ATG12* 3′UTR with or without five point mutations with a luciferase reporter. Co-transfection with a miR-200b mimic markedly inhibited luciferase activity in the reporter vector containing the wild-type *ATG12* 3′UTR but not the mutant 3′UTRs in both SPC-A1/DTX and HEK-293 cells (Fig. 2B and Supplementary Fig. 3). Consistent with these findings, docetaxel-resistant cells, including SPC-A1/DTX and H1299/DTX cells, had higher basal ATG12 mRNA and protein levels compared with their parental cells (Fig. 2C). Additionally, overexpression of miR-200b decreased ATG12 mRNA and protein levels in both SPC-A1/DTX and H1299/DTX cells, whereas silencing endogenous miR-200b increased ATG12 expression in parental cells (Fig. 2D and Supplementary Fig. 1C). Similar to miR-200b overexpression, silencing ATG12 prevented both LC3-II accumulation and P62 degradation in docetaxel-resistant cells (Fig. 2E).

RETRACTED

**Figure 2:** MiR-200b inhibits autophagy by directly targeting ATG12 **A.** Predicted miR-200b consensus sequences in the ATG12 3′UTR. **B.** Luciferase activity analysis of ATG12 3′UTR (wild type and mutant constructs) were performed after co-transfection with PmiR-200b in HEK-293 cells by using the Dual-luciferase Reporter Assay System. The data are expressed as the mean ± SD (*n* = 3). *P < 0.05 vs the PmiR-NC. **C.** Western blot and qRT-PCR was used to analyze the expression of ATG12 in both parental and docetaxel-resistant cells. ATG12/GAPDH ratios were calculated using Image J densitometric analysis (three independent experiments gave similar results). **D.** SPC-A1 cells and H1299 cells were transfected with AmiR-200b or AmiR-NC whereas SPC-A1/DTX cells and H1299/DTX cells were transfected with PmiR-200b or PmiR-NC. ATG12 expression was determined by western blot and qRT-PCR analysis. ATG12/GAPDH ratios were calculated using Image J densitometric analysis. Data are represented as mean ± SD of three independent experiments. *P < 0.05, **P < 0.01. **E.** SPC-A1/DTX cells and H1299/DTX cells were transfected with ATG12 siRNA, followed by treatment with docetaxel (100 μg/L) or cisplatin (1.5 μg/ml). LC3, P62 and ATG12 expression levels were evaluated by western blot. LC3-II/LC3-I, P62/GAPDH and ATG12/GAPDH ratios were calculated using Image J densitometric analysis (three independent experiments gave similar results). **F.** Western blot for LC3, p62 and ATG12 of whole lysates of SPC-A1/DTX cells and H1299/DTX cells transfected with PmiR-200b, pDsRed1 ATG12 or both. LC3-II/LC3-I, P62/GAPDH and ATG12/GAPDH ratios were calculated using Image J densitometric analysis (three independent experiments gave similar results). **G.** SPC-A1/DTX cells and H1299/DTX cells were co-transfected with GFP-LC3 plasmids and PmiR-200b, pDsRed1 ATG12 or both combinations (bar: 50 μm). Data are represented as mean ± SD of three independent experiments. *P < 0.05; **P < 0.01.

As a final confirmation of the inhibitory effect of miR-200b on ATG12, we performed rescue experiments by overexpressing ATG12 in SPC-A1/DTX and H1299/DTX cells, which largely negated miR-200b-dependent autophagy suppression, as demonstrated by elevated LC3-II expression, which approached the level in control cells, and the increased percentage of GFP-positive cells (Fig. 2F, 2G). Taken together these results demonstrate that *ATG12* is a direct target of miR-200b.

RETRACTED

### MiR-200b inhibits starvation and rapamycin-induced autophagy

We next investigated the role of miR-200b on commonly recognized autophagy stimuli. Exposing cells to nutrient starvation (using Hank's balanced salt solution), caused a decrease in endogenous miR-200b expression after 1 hour, and a delayed response in increased *ATG12* mRNA expression, which returned to near basal levels about 4 hours after the addition of exogenous miR-200b to SPC-A1 cells (Fig. 3A). Similar results were obtained in H1299 cells (Supplementary Fig. 4A). Enhanced *ATG12* expression corresponded with decreased miR-200b expression, implying that an early decrease in miR-200b expression may regulate the magnitude of *ATG12* gene expression. Consistently, overexpressing miR-200b or a specific siRNA that targets *ATG12* inhibited starvation-induced conversion of LC3-I to LC3-II, prevented p62 degradation and reduced the number of punctate GFP-positive cells (Fig. 3B, 3C and Supplementary Fig. 4B, 4C).

**Figure 3:** MiR-200b inhibits starvation and rapamycin-induced autophagy in SPC-A1 cells **A.** SPC-A1 cells were incubated in HBSS for different time periods (0 to 8 h). Exogenous miR-200b was transfected into cells at 4 h. The relative expression levels of miR-200b mRNA and ATG12 mRNA were assessed by qRT-PCR, with expression in the control set as 1.0. **B, D.** SPC-A1 cells were transfected with PmiR-200b, ATG12 siRNA or NC, followed by treatment with B. HBSS for 4 h or D. rapamycin (50 nM) for 2 h. The protein levels of LC3, P62 and ATG12 were assayed by western blot. LC3-II/LC3-I, P62/GAPDH and ATG12/GAPDH ratios were calculated using Image J densitometric analysis (three independent experiments gave similar results). **C, E.** SPC-A1 cells were co-transfected with either PmiR-200b or ATG12 siRNA and GFP-LC3 plasmid, and then exposed to C. HBSS for 4 h or E. rapamycin (50 nM) for 2 h. Data are shown as mean ± SD of three replicates and are representative of three independent experiments. *P < 0.05; **P < 0.01. **F.** Western blot analysis detected the expression of LC3 and P62 in AmiR-200b-transfected SPC-A1 cells after treatment with rapamycin (50 nM) for 2 h. LC3-II/LC3-I and P62/GAPDH ratios were calculated using Image J densitometric analysis (three independent experiments gave similar results).

We next examined the effect of miR-200b on autophagy induced by another stimulus, the mTOR blocker rapamycin [19]. Suppression of mTOR activity activates the Ulk1/2 complex, an early event during autophagy, although mTOR-independent pathways also exist [20]. In line with the starvation data, addition of rapamycin accelerated GFP-LC3 punctate formation, LC3-II turnover as well as p62 clearance, but these results were attenuated after transfection with either PmiR-200b or Atg12 siRNA (Fig. 3D, 3E and Supplementary Fig. 4D, 4E). ATG12 protein levels were reduced in both parental cells overexpressing miR-200b, both in the presence or absence of rapamycin. In addition, combined treatment with rapamycin and AmiR-200b transfection had a cumulative effect on ATG12 and LC3-II expression (Fig. 3F and Supplementary Fig. 4F). Hence, miR-200b regulates both starvation- and rapamycin-induced autophagy.

RETRACTED

### MiR-200b increases chemosensitivity of LAD cells by targeting *ATG12 in vitro*

Based on the finding that miR-200b was the most greatly downregulated miRNA in SPC-A1/DTX cells compared with parental SPC-A1 cells, we sought to evaluate whether miR-200b-induced chemosensitivity was dependent on ATG12 suppression. Restoration of miR-200b or *ATG12* knockdown caused cell death and suppressed growth of SPC-A1/DTX and H1299/DTX cells, as shown by MTT and colony formation assays, respectively (Fig. 4A, 4B and Supplementary Fig. 5A, 5B). Notably, the PmiR-200b-dependent cytotoxic effects of docetaxel and cisplatin were eliminated by ectopic expression of ATG12. Consistent with these data, a loss-of-function study verified that AmiR-200b limited the cell killing efficiency and promoted colony-formation efficiency of these agents in SPC-A1 and H1299 cells, but that these events were reversed by *ATG12* silencing (Fig. 4C, 4D and Supplementary Fig. 5C, 5D).

**Figure 4:** MiR-200b increases chemosensitivity of SPC-A1/DTX cells by targeting ATG12 **A, B.** SPC-A1/DTX cells were transfected with PmiR-200b, pDsRed1 ATG12, or both or with ATG12 siRNA, followed by exposure to indicated doses of docetaxel or cisplatin for 48 h. A. MTT assay showing cell viability; B. colony formation assay showing cell proliferation. **C, D.** SPC-A1 cells were transfected with AmiR-200b, ATG12 siRNA or both, and then treated with the indicated concentrations of docetaxel or cisplatin for 48 h. C. MTT assay showing cell viability; D. colony formation assay showing cell proliferation. Data are shown as mean ± SD of three replicates and are representative of three independent experiments. *P < 0.05; **P < 0.01.

Next we determined the effect of miR-200b on apoptosis. Compared with the control group, miR-200b overexpression resulted in increased apoptosis of docetaxel-resistant cells when exposed to cytotoxic agents, as indicated by an enhanced percentage of Annexin V-stained cells and a massive cleavage of PAPR and caspase-3 (Fig. 5A, 5B and Supplementary Fig. 6A, 6B). However, ectopic expression of ATG12 largely abrogated both docetaxel and cisplatin-induced apoptotic cell death due to activation of autophagy. Meanwhile, transfection of SPC-A1 and H1299 cells with the miR-200b inhibitor substantially diminished drug-induced apoptosis (Fig. 5C, 5D and Supplementary Fig. 6C, 6D). Taken together, these data indicate that miR-200b enhances the chemosensitivity of LAD cells in an ATG12-dependent manner.

RETRACTED

**Figure 5:** MiR-200b increases the sensitivity of SPC-A1/DTX cells to apoptosis by targeting ATG12 **A, B.** SPC-A1/DTX cells were transfected with PmiR-200b, pDsRed1 ATG12, or both, or with ATG12 siRNA, followed by exposure to docetaxel (100 μg/L) or cisplatin (1.5 μg/ml) for 48 h. Apoptosis was measured by A. flow cytometry with Annexin-V staining (Data are expressed as mean ± SD of three independent experiments. *P < 0.05; **P < 0.01); and B. western blotting was performed for apoptosis markers (c-caspase-3 and c-PARP). C-caspase3/caspase3, c-PARP/PARP and ATG12/GAPDH ratios were calculated using Image J densitometric analysis (three independent experiments gave similar results). **C, D.** SPC-A1 cells were transfected with AmiR-200b, ATG12 siRNA or both, and then treated with docetaxel (20 μg/L) or cisplatin (0.8 μg/ml) for 48 h. Apoptosis was measured by C. flow cytometry with Annexin-V staining (Data are expressed as mean ± SD of three independent experiments. *P < 0.05; **P < 0.01.); and D. western blot for apoptosis markers (c-caspase-3 and c-PARP). C-caspase3/caspase3, c-PARP/PARP and ATG12/GAPDH ratios were calculated using Image J densitometric analysis (three independent experiments gave similar results).

### MiR-200b enhances the antitumor efficacy of docetaxel *in vivo*

To investigate the effect of miR-200b on docetaxel sensitivity of LAD *in vivo*, SPC-A1/DTX cells were stably transfected with a miR-200b plasmid construct (pcDNA/miR-200b) or control plasmid (pcDNA/miR-NC) and subcutaneously inoculated into nude mice. Tumor-bearing mice were treated with docetaxel at a dose of 1 mg/kg every other day with three doses in total and tumor volumes were monitored daily. Tumors derived from pcDNA/miR-200b-transfected SPC-A1/DTX cells were substantially smaller than the control group. Remarkably, SPC-A1/DTX-derived tumor outgrowth was prevented when docetaxel treatment was administered in a miR-200b-overexpressed genetic background (Fig. 6A, 6B). Immunohistochemistry and western blot analysis of the tumor specimens confirmed diminished ATG12 expression and decreased autophagy activity in pcDNA/miR-200b-transfected tumors in response to docetaxel when compared with pcDNA/miR-NC-transfected tumors (Fig 6B, 6C). TUNEL staining of xenografts showed higher apoptosis in the pcDNA/miR-200 group than in the control group following treatment with docetaxel (Fig. 6C). Conversely, ki67 (a marker of cell proliferation [21]) was clearly diminished in pcDNA/miR-200b-transfected tumors (Fig. 6C). These observations provide further evidence for the role of miR-200b in determining the response of NSCLC cells to docetaxel *in vivo*.

RETRACTED

**Figure 6:** MiR-200b enhances the antitumor efficacy of docetaxel *in vivo* **A.** Nude mice were subcutaneously injected with 5 × 10^6^ cells stably transfected with pcDNA miR-200b or pcDNA miR-NC and treated with docetaxel (1mg/kg) beginning at day eight. Tumor size was measured every 2 days after docetaxel treatment (*n* = 3, *P < 0.05). **B.** Representative photographs of tumors formed at 16 days after subcutaneous transplantation are displayed. **C.** Hematoxylin and eosin (H&E)-stained, ATG12-stained, ki67-stained and TUNEL staining in paraffin sections of the tumors. **D.** Western blot analysis of LC3 and ATG12 in implanted tumors. Data shown are representative of three identical experiments. LC3-II/LC3-I and P62/GAPDH ratios were calculated using Image J densitometric analysis (three independent experiments gave similar results).

### Downregulation of miR-200b correlates with upregulation of ATG12, decreased sensitivity to docetaxel and poor prognosis in lung adenocarcinoma tissues

To further investigate the relationship between miR-200b and ATG12 expression *in vivo*, tissue samples were obtained from 60 clinical LAD cases from patients diagnosed with advanced lung adenocarcinoma. Samples were classified as “sensitive” or “insensitive” depending on the responses to docetaxel-based chemotherapies. According to the data in Fig. 7A, miR-200b mRNA expression was markedly decreased in the “insensitive” group compared with the “sensitive” group, and vice versa in the case of *ATG12* mRNA expression. ATG12 protein expression was similarly decreased in the “sensitive” tumor tissues, as measured by immunohistochemical staining (Fig. 7B). This inverse association between miR-200b and ATG12 expression was significant based on linear regression analysis (Fig. 7C). LAD tissue samples were next categorized as miR-200b-high or -low using the median miR-200b mRNA expression level as threshold (median = 1.86, normalized to U6 snRNA). Low miR-200b expression was significantly correlated with advanced clinical stage and poor response to docetaxel-based chemotherapy (Fig. 7D).

**Figure 7:** Downregulation of miR-200b expression correlates with upregulation of ATG12 expression, decreased sensitivity to docetaxel and poor prognosis in lung adenocarcinoma tissues **A.** qRT-PCR was performed to analyze the relative mRNA expression of miR-200b and ATG12 in docetaxel-sensitive (*n* = 27) and insensitive (*n* = 33) LAD tissues. MiR-200b and ATG12 mRNA abundances were normalized to U6 RNA and GAPDH, respectively. **B.** Protein expression of ATG12 was determined by immunochemical staining (magnification 200×). **C.** Expression levels of miR-200b and ATG12 mRNA were inversely correlated among tissue samples as measured by linear regression analysis. **D.** The Kaplan–Meier survival curve shows that patients with high miR-200b expression have shorter progression-free survival (PFS) than those with low miR-200b expression (log-rank test, *P* = 0.021). Data are expressed as mean ± SD of three independent experiments. *P < 0.05.

RETRACTED

The association of miR-200b expression with patient survival was further analyzed. Patients with a low miR-200b expression (*n* = 34) had a shorter progression free survival (PFS) than those patients with high miR-200b expression (*n* = 26; median: 3.4 months vs. 4.4 months). Therefore, these data strongly suggest that decreased miR-200b expression, which is inversely correlated with ATG12 expression in LAD patients, is linked to poor prognosis (Table 1).

**Table 1:** Correlation between miR-200b expression and clinicopathological factors of LAD patients

Variables	MiR-200b expression		*P* value
	low (*n* = 34)	high (*n* = 26)	
**Gender**			0.455
Female	19	12	
Male	15	14	
**Age (years)**			0.930
<60	14	11	
≥60	20	15	
**Smoking condition**			0.660
Nonsmokers	15	10	
Smokers	19	16	
**Tumor differation**			0.228
Well+Moderate	13	14	
poor	21	12	
**Clinical stage**			0.021*
IIIB	12	17	
IV	22	9	
**Tumor response**			0.024*
CR+PR	11	16	
SD+PD	23	10	

* *p* < 0.05.

## DISSCUSSION

Autophagy is considered to play a dual role in the regulation of cell fate decision in the context of cancer treatment [22]. Numerous studies have focused on the association between the cytoprotective effects of autophagy and the development of chemoresistance. Several autophagy inhibitors are now in clinical trials [23]. Importantly, miRNAs are frequently dysregulated in chemo- or radio-resistant cancers, where they have been shown to target autophagy-related genes or modulators [24–26]. Based on our previously reported miRNA microarray-based profile between docetaxel-sensitive SPC-A1 cells and resistant SPC-A1/DTX cells, we hypothesized that the differentially expressed miRNAs are associated with docetaxel resistance, with miR-200b being the most significantly down-regulated miRNA in SPC-A1/DTX cells. Here, we show that introduction of exogenous miR-200b into SPC-A1/DTX cells suppressed autophagy activity and resensitized cells to chemotherapy. Inversely, silencing endogenous miR-200b induced autophagy in SPC-A1 cells and increased resistance to chemotherapy. These results reveal a tight relationship between miR-200b and autophagy activation in LAD.

RETRACTED

The miR-200 family is aberrantly expressed in a variety of cancers [27, 28], and regulates multiple pathway components including a number of transcription factors involved in tumor migration and invasion [29] [30]. In the present study, we uncovered a novel role for miR-200b in autophagy regulation and identified *ATG12* as a direct miR-200b target. In LAD cells, endogenous miR-200b was downregulated in response to cellular stress caused by starvation and rapamycin, followed by upregulation of ATG12. Downregulation of miR-200b upon autophagy stimulation might remove translational inhibition on *ATG12* and subsequently promote autophagosome formation. However, further introduction of exogenous miR-200b greatly decreased ATG12 expression and blocked starvation and rapamycin-induced autophagy.

ATG12 is a key component in autophagosome formation and is upregulated in trastuzumab-unresponsive breast cancer cells [31] and radioresistant pancreatic cancer cells [32]. Our work shows that ATG12 is also upregulated in docetaxel-resistant LAD cells. Both ATG12 silencing and miR-200b overexpression significantly sensitized SPC-A1/DTX and H1299/DTX cells to docetaxel and cisplatin.

In an *in vivo* setting, miR-200b overexpression drastically attenuated ATG12 expression and subsequent autophagy activity, preventing long-term tumor cell survival by exposing them to metabolic stress and suppressing eventual tumor regrowth following docetaxel treatment. Consistent with these findings, miR-200b was inversely correlated with ATG12 in clinical docetaxel-treated LAD tissue samples. Specifically, a relative increase in miR-200b coupled with a decrease in ATG12 expression was observed in tissue samples from docetaxel-sensitive patients. Moreover, patients with relatively lower levels of miR-200b expression had poorer prognosis. Taken together, our data therefore provide, for the first time, evidence that miR-200b could significantly affect LAD chemosensitivity through negative regulation of autophagy-related genes (Fig. 8).

**Figure 8:** Mechanism whereby miR-200b modulates ATG12-dependent chemoresistance MiR-200b inhibits ATG12 expression, which leads to a decrease in autophagy that contributes to chemoresistance.

Interestingly, another miRNA, miR-23b, has also been reported to target *ATG12* with different 3′UTR sequences (bases 172–178 and 1281–1288) than miR-200b (bases 946–952) [32]. Considering the imperfect match and relatively short base pair seed sequence characteristic of miRNA–mRNA interactions, it is not surprising that a single miRNA can concurrently target multiple genes while a single mRNA may have multiple miRNA target sites [33].

RETRACTED

Apart from ATG12, there are over 35 other autophagy-related gene products and autophagy-regulating factors [7]. For instance, we previously reported that the autophagy modulator HMGB1 promotes formation of the Beclin-1-PI3K-III complex by activating the MEK/ERK1/2 signaling pathway, thereby accelerating autophagosome nucleation [12]. A recent study suggests that miR-34a may modulate *HMGB1* gene expression and subsequent autophagic response [34]. However, we did not find a putative miR-200b-binding site within the 3′UTR of *HMGB1* or significant changes in *HMGB1* levels when modulating miR-200b expression (Data not shown). The miR-200b-ATG12 and HMGB1-MEK/ERK1/2-Beclin1/PI3K-III pathways seem to be concurrently implicated in autophagic abnormalities of LAD cells. Further studies are warranted to elucidate the relationship between these two mechanisms in order to expand our understanding of autophagy.

Taken together, the present work demonstrates for the first time that miR-200b could decrease autophagy activity and increase chemotherapy-induced cell death by targeting *ATG12* in LAD cells. Therefore, targeting miR-200b-ATG12 signaling may be a potential strategy for reversing chemoresistance in combating LAD.

## MATERIALS AND METHODS

### Cell lines and reagents

Human lung adenocarcinoma SPC-A1 and H1299 cells were purchased from the Tumor Cell Bank of the Chinese Academy of Medical Science (Shanghai, China) and cultured in RPMI 1640 medium containing 10% fetal bovine serum, ampicillin and streptomycin at 37°C in a humidified atmosphere (95% air and 5% CO_2)_. Docetaxel-resistant SPC-A1 and H1299 cell lines (SPC-A1/DTX and H1299/DTX) were established and preserved in a final concentration of 50 μg/L docetaxel. Antibodies against GAPDH, LC3, p62, caspase3, activated (cleaved) caspase-3 (c-caspase-3), PARP, cleaved PARP (c-PARP), ATG5, ATG12 were purchased from Cell Signaling Technology. Bafilomycin A1 and 3-MA were obtained from Sigma Aldrich (St. Louis, MO).

### cDNA constructs, siRNA and transfection

The GFP-tagged LC3 cDNA expression construct was a gift from Dr. Noboru Mizushima (Tokyo Medical and Dental University, Tokyo, Japan). The miRNA mimics, miRNA inhibitors, ATG5 siRNA, ATG12 siRNA, pDsRed1 Atg12 were synthesized by GenePharma (Shanghai, China). Cells were transfected using Lipofectamine 2000 (Invitrogen, USA), according to the manufacturer's protocol.

### Cell viability

Cells were seeded into 96-well plates (3 × 10^3^ cells/well) directly or 24 h after transfection. After treatment with the indicated drug combinations for 48 h, cell viability was assessed via 3-(4,5-dimethylthiazol-2-yl)-2, 5-diphenyl-trtrazolium bromide (MTT) assay as described previously [35].

RETRACTED

### Colony formation assay

Forty-eight hours after transfection, cells were exposed to various treatments, and then seed into 6-well plates. Cells were allowed to adhere and grow for between 10 to 14 days. To visualize colonies, cells were fixed with methanol and stained with 0.1% crystal violet. Colonies with ≥50 cells were manually counted under a dissection microscope.

### Western blot analysis

Cells were washed with PBS, harvested in ice-cold PBS and centrifuged at 2000 rpm at 4°C. Cells were placed for 30 min on ice in RIPA buffer in the presence of a cocktail proteinase inhibitor (Sigma-Aldrich, USA). The protein lysate was separated by SDS-PAGE, transferred onto PVDF membranes (Millipore, USA), and analyzed as described previously [15].

### Real-time quantitative PCR (qRT-PCR) analysis

Total RNA was extracted with Trizol (Takara, Japan) reagent and concentrations were measured by a spectrophotometer. Reverse transcription and qRT-PCR were conducted using SYBR PrimeScript™ miRNA RT-PCR kit (Takara, Japan, Cat. No. RR716) according to the manufacturer's instructions. The conditions for PCR reactions were: 95°C for 30 s followed by 40 cycles of 95°C for 5 s and 60°C for 30 s, using a StepOnePlus™ thermal cycler. MiRNA expression levels were normalized to *U6* RNA. SYBR Premix Ex Taq (Takara, Japan, Cat. No. RR420A) was also used to detect mRNA. SYBR Green quantitative PCR amplifications were performed on a StepOnePlus™ thermal cycler, in 25 μl volumes containing 12.5 μl of 2 × SYBR Green PCR Master Mix. The thermal profile for real-time PCR was: 95°C for 30 s; followed by 40 cycles of 95°C for 5 s, 60°C for 30 s and 70°C for 30 s. Relative mRNA expression was normalized to GAPDH using the comparative ΔΔC_T_ method; values are expressed as 2^−ΔΔCT^. Primer sequences are listed in Supplementary Table 1.

### Apoptosis assay

We measured apoptosis using an Annexin-V-fluorescein isothiocyanate apoptosis detection kit (Oncogene Research Products, Boston, MA) that quantitatively measures percentages of early apoptotic cells via flow cytometry. Western blot analyses for c-PARP and c-caspase-3 after various treatments were also performed. The degree of apoptosis in tissues was assessed with the TUNEL kit (Roche) according to the manufacturer's instructions.

### Dual luciferase reporter assay

Cells were lysed in passive lysing buffer and then analyzed for firefly and Renilla luciferase activities using the commercial Dual-Luciferase reporter assay system (Promega, E1910) according to the manufacturer's instructions. Firefly luciferase activity was normalized to the Renilla luciferase activity.

RETRACTED

### GFP-LC3 analysis

Forty-eight hours after GFP-LC3 transfection, cells were fixed in 3.7% formaldehyde for 20 min, washed with PBS, mounted in glycerol in PBS and inspected using a fluorescence microscope. Cells with ≥10 GFP-LC3 dots were considered positive. At least 150 GFP positive cells were counted under each condition, and the graphs were plotted as percentage of GFP-LC3 dot positive cells divided by the total GFP-positive cell population.

### Transmission electron microscopy

Cells harvested by trypsinization were fixed in 2.5% glutaraldehyde plus 4% paraformaldehyde in 0.1 M phosphate buffer, and then post-fixed in 1% tetroxide buffer. After dehydration in a graded series of acetone, cells were embedded in spur resin. Thin sections were cut on a Reichert Ultracut E microtome. Sectioned grids were stained with saturated solution of uranyl acetate and lead citrate.

### Mice xenograft models and immunohistochemistry analysis

Animal maintenance and experimental procedures were strictly performed following the guidelines of the Institutional Review Board and approved by the Ethics Committee of Jinling Hospital. Approximately 5 × 10^6^ SPC-A1/DTX/pcDNA miR-200b or SPC-A1/DTX/miR-NC cells were subcutaneously transplanted into twelve 6-week-old BALB/c mice (six mice for SPC-A1/DTX/pcDNA miR-200b cells, and six for SPC-A1/DTX/miR-NC cells). Tumor volumes were examined every other day and were calculated using the equation: V = A × B^2^/2(mm^3^), where A is the largest diameter and B is the perpendicular diameter. When the average tumor size reached approximately 100 mm^3^, docetaxel was administered via intraperitoneal injection at a dose of 1 mg/kg at one dose every other day for a total of three doses. In each of the group transplanted with SPC-A1/DTX/pcDNA miR-200b cells or SPC-A1/DTX/miR-NC cells, three mice were injected with docetaxel and three were injected with 0.9% normal saline as control. All mice were sacrificed 16 days later, and the tumors were dissected out. The primary tumors were excised and analyzed by hematoxylin and eosin (H&E) staining, immunohistochemistry staining of proliferating cell nuclear antigen (PCNA), ATG12, TUNEL staining and western blot analysis for LC3 and ATG12 protein expression.

### Tissue samples

A total of 60 lung adenocarcinoma cancer tissues were obtained from the Department of Cardiothoracic Surgery, Jinling Hospital between 2006 and 2010. The study was approved by the Ethics Committee of Jinling Hospital. All patients met the following criteria: a histological diagnosis of primary LAD with at least one measurable lesion; clinical stage IIIB–IV; first-line chemotherapy with either docetaxel 75mg/m^2^ and cisplatin 100 mg/m^2^ or docetaxel 75 mg/m^2^ and carboplatin (area under the curve 6mg/mL/min) administered every 3 weeks for a maximum of six cycles; availability of sufficient tumor tissue in paraffin blocks for assessment by immunohistochemistry. Tumor response was examined by computed tomography and evaluated according to the Response Evaluation Criteria in Solid Tumors (RECIST) as complete response (CR), partial response (PR), stable disease (SD), or progressive disease (PD). Based on the above response evaluation criterion, tumor samples were divided into “sensitive” (CR or PR) and “insensitive” (SD or PD) groups.

RETRACTED

### Statistical analysis

Data are expressed as mean ± SD of ≥ three separate experiments. SPSS17.0 software was used for statistical analysis. Multiple group comparisons were analyzed with one-way ANOVA; two-group comparisons were performed with Student's *t* test. Survival probabilities were determined using Kaplan–Meier analyses and compared by the log-rank test. *P* < 0.05 was considered statistically significant.

## SUPPLEMENTARY FIGURES AND TABLE



## Abbreviations

NSCLC: non-small cell lung cancer
LAD: lung adenocarcinoma
MAP1LC3: microtubule-associated protein1 light chain 3
PE: phosphatidylethanolamine
miRNAs: microRNAs
3′-UTR: 3′-untranslated regions
HMGB1: high-mobility group box 1
Baf A1: Bafilomycin A1.
